This article has been retracted.

# The Effect of lncRNA SNHG3 Overexpression on Lung Adenocarcinoma by Regulating the Expression of miR-890

**DOI:** 10.1155/2021/1643788

**Published:** 2021-07-08

**Authors:** Baojie Kang, Caihong Qiu, Ying Zhang

**Affiliations:** ^1^Department of Respiratory, Weifang Yidu Central Hospital, Weifang City, Shandong, China; ^2^Department of ICU, Zibo Central Hospital, Zibo City, Shandong, China

## Abstract

The lncRNA small nucleolar host gene 3 (SNHG3) was discovered to play an important role in the occurrence and development of lung adenocarcinoma (LUAD). However, the underlying molecular mechanism of SNHG3 in LUAD remains unclear. In the present study, SNHG3 expression levels in LUAD tissues and cell lines were analyzed using reverse transcription-quantitative PCR. The effects of SNHG3 on the proliferation, apoptosis, migration, and invasion of LUAD cells were determined using Cell Counting Kit-8, colony formation, flow cytometry, wound healing, and Transwell chamber assays, respectively. The specific underlying mechanism of SNHG3 in LUAD was investigated using bioinformatics analysis and a dual luciferase reporter assay. The results revealed that SNHG3 expression levels were downregulated in LUAD tissues and cell lines. Functionally, SNHG3 overexpression suppressed the proliferation, migration, and invasion of LUAD cells, while promoting apoptosis. Mechanistically, microRNA- (miR-) 890 was identified as a potential target of SNHG3, and its expression was negatively regulated by SNHG3. Notably, SNHG3 was found to promote LUAD progression by targeting miR-890. In conclusion, the findings of the present study revealed that lncRNA SNHG3 promoted the occurrence and progression of LUAD by regulating miR-890 expression.

## 1. Introduction

Lung cancer is a common type of cancer with high incidence and mortality rates worldwide [1]. Non-small-cell lung cancer (NSCLC) represents ∼85% of all lung cancer types and has a mortality rate of ∼50%. Lung adenocarcinoma (LUAD), a leading cause of cancer-related mortality, accounts for ∼40% of NSCLCs and has a 5-year survival rate of only 15% [2]. At present, patients with LUAD are usually diagnosed at the terminal stage or following metastasis due to the lack of effective biomarkers and obvious early symptoms [3, 4]. For more than half a century, even with the significant progress and development made in molecular biology, oncology, and medicinal technology, the treatment of LUAD has been and remains ineffective [5]. In addition, although a large number of molecular biology studies have focused on investigating the mechanisms underlying LUAD, the exact molecular mechanism of LUAD remains unclear. Thus, further investigations to identify LUAD-associated pathogenic genes and the underlying molecular mechanisms of LUAD are required.

Long noncoding RNAs (lncRNAs), which are functional transcripts of >200 nucleotides in length, have been discovered to serve important roles in modulating the pathological and physiological progression of numerous cancer types [6–9]. Accumulating studies have reported that the abnormal expression of lncRNAs was associated with the progression of different malignant tumor types, including breast cancer [9], prostate cancer [10], liver cancer [11], and LUAD [12, 13]. Numerous lncRNAs, such as metastasis-associated lung adenocarcinoma transcript 1 [12], long intergenic non-protein-coding RNA 1512 [13], MIR31 host gene [14], FEZ family zinc finger 1 antisense RNA 1 [15], and urothelial cancer associated 1 [16], were found to be closely associated with LUAD occurrence and development. In addition, the lncRNA DiGeorge syndrome critical region gene 5 was reported to promote the progression of LUAD by downregulating microRNA- (miRNA/miR-) 22-3p expression [17]. The lncRNA small nucleolar host gene 3(SNHG3) is a long noncoding RNA. At present, its potential role and mechanism in lung adenocarcinoma have not been reported. SNHG3, also known as the host gene of U17 (U17HG), is located in band 6 in region 3 of the short arm of chromosome 1. The lncRNA small nucleolar host gene 3 (SNHG3) has been demonstrated to serve a role in multiple types of cancer. In fact, an increasing number of studies have revealed that the expression levels of SNHG3 were upregulated in numerous tumor types, and SNHG3 upregulation markedly promoted tumor cell proliferation, migration, and invasion, thereby indicating that SNHG3 may represent a novel oncogenic lncRNA [18]. For example, SNHG3 promoted the migration and invasion of osteosarcoma cells by regulating the miR-151a-3p/RAB22A, member RAS oncogene family axis [19]. In NSCLC, SNHG3 promoted the proliferation, migration, and invasion of NSCLC cells by activating the TGF-*β* and IL-6/JAK2/STAT3 signaling pathways [20]. These studies suggested that SNHG3 may serve a role as a novel oncogene in numerous cancer types. Nevertheless, the specific regulatory mechanism of SNHG3 in LUAD requires further study.

The current study hypothesized that SNHG3 may promote LUAD occurrence and development by targeting miR-890 expression. Thus, the expression levels of SNHG3 and miR-890 in LUAD tissues and cell lines were analyzed. The potential functions of SNHG3 and its association with miR-890 were also investigated *in vitro*. The results of the present study may provide a novel insight into potential targets for the treatment of LUAD.

## 2. Materials and Methods

### 2.1. Patient Studies

LUAD and adjacent normal tissues were obtained from 66 patients with LUAD (men and women account for 50%, respectively) who were diagnosed at Weifang Yidu Central Hospital (China). Included patients had neither received surgery nor chemotherapy prior to sample collection. The present study was approved by the Ethics Committee of Weifang Yidu Central Hospital, and all enrolled patients provided written informed consent. All tissues were stored at –80°C before use.

### 2.2. Cell Lines and Culture

The human normal lung epithelial cell line, 16HBE, and human LUAD cell lines (A549, H1299, and H1975) were obtained from the Cell Bank of Type Culture Collection of the Chinese Academy of Sciences. All cells were cultured in DMEM (Nanjing KeyGen Biotech Co., Ltd.) and maintained in a humidified atmosphere with 5% CO_2_ at 37°C.

### 2.3. Cell Transfection

The pcDNA 3.1 and pcDNA3.1 SNHG3 plasmids, negative control (NC) inhibitor, miR-890 inhibitor, NC mimic, and miR-890 mimic were purchased from Invitrogen; Thermo Fisher Scientific, Inc. The synthetic oligonucleotides or plasmids were transfected into cells using Lipofectamine^®^ 2000 (Invitrogen; Thermo Fisher Scientific, Inc.).

### 2.4. Cell Counting Kit-8 (CCK-8) Assay

The cells were gently seeded at a density of 1 × 106 cells/well into 96-well plates by the experimenter. Following 24, 48, 72, 96, or 120 h of culture, the CCK-8 reagent (Beyotime Institute of Biotechnology) was added to each well. The cell density was measured at a wavelength of 450 nm.

### 2.5. Colony Formation Assay

The transfected cells were seeded into a 6-well plate and cultured for 14 days; during this process, the medium was replaced every 2 days. Following the incubation, the formed colonies were fixed with 4% formaldehyde and stained with crystal violet (Sangon Biotech Co., Ltd.) for 3 min to visualize the colonies, which were defined as >50 cells. The colony formation rate was calculated using the following equation: colony formation rate (%) = (number of colonies/number of seeded cells) × 100.

### 2.6. Reverse Transcription-Quantitative PCR (RT-qPCR)

Total RNA was extracted from LUAD cell lines and tissues using TRIzol® reagent (Invitrogen; Thermo Fisher Scientific, Inc.). Total RNA was reverse transcribed into cDNA using a PrimeScript RT reagent kit (Qiagen, Inc.). qPCR was subsequently performed using SYBR Green (Takara Bio, Inc.), with U6 as the control gene. The following primer pairs were used for the qPCR: SNHG3 forward, 5′-TTCAAGCGATTCTCGTGCC-3′ and reverse, 5′-AAGATTGTCAAACCCTCCCTGT-3′; miR-890 forward, 5′-CGGCTTCCTGTGCTAAGCGT-3′ and reverse, 5′- AACGCTTCACGAATTTGCGT-3′; and U6 forward, 5′-CTCGCTTTCGGCAGCACA-3′ and reverse, 5′-AACGCTTCACGAAATTTGCGT-3′.

### 2.7. Cell Apoptosis Assay

Following trypsinization and centrifugation, 1 × 10^6^ cells were collected and incubated with 500 *μ*l buffering agent containing Annexin V-FITC and PI in the dark for 30 min. The cell apoptotic rate was analyzed using flow cytometry (Beckman Coulter, Inc.).

### 2.8. Wound Healing Assay

The migratory ability of LUAD cells was analyzed using a wound healing assay. Briefly, 1 × 10^6^ transfected cells were cultured for 24 h, and upon reaching confluence, a straight line was scratched into the cell monolayer to generate an artificial wound. The area of the scratch was visualized under a microscope at 0 and 48 h and analyzed using an image analysis and detection system.

### 2.9. Cell Invasion Assay

The invasive ability of LUAD cells was measured using Transwell plates (8.0 µm pores; Nanjing KeyGen Biotech Co., Ltd.). Briefly, 1 × 10^6^ cells/well were seeded into the upper chamber of the Transwell plates. Following 48 h of incubation, the invasive cells were fixed and stained with crystal violet. Stained cells were visualized and semiquantified using a microscope (Nikon Corporation).

### 2.10. Dual Luciferase Reporter Assay

Wild-type (WT) or mutant (Mut) SNHG3 3′-untranslated region (UTR) fragments containing the miR-890 binding sites were synthesized and inserted into the pGL3-basic plasmid (Promega Corporation) to construct SNHG3-WT or SNHG3-Mut reporter vectors, respectively. LUAD cells were cotransfected with the aforementioned reporter vectors and miR-890 inhibitor or NC inhibitor. Following 48 h of transfection, the relative luciferase activity was measured using a Dual Luciferase Reporter assay system (Promega Corporation).

### 2.11. Statistical Analysis

Statistical analysis was performed using SPSS 19.0 software (IBM Corp.), and data are presented as the mean ± SD. Statistical differences between two or more groups were performed using Student's *t*-test or one-way ANOVA, respectively. Kaplan–Meier survival analysis was used to evaluate the association between the overall survival of patients with LUAD and SNHG3 expression levels. The Gene Expression Profiling Interactive Analysis (GEPIA) database was used to analyze the survival of patients with either low or high expression of SNHG3. *P* < 0.05 was considered to indicate a statistically significant difference.

## 3. Results

### 3.1. SNHG3 Expression Levels Are Downregulated in LUAD Tissues and Cell Lines

To determine the potential regulatory roles of SNHG3 in LUAD, RT-qPCR analysis was performed. The clinicopathological characteristics of patients are shown in Table 1. SNHG3 expression levels were downregulated in LUAD tissues compared with adjacent normal tissues (Figure 1(a)). The results of the Kaplan–Meier analysis revealed that patients with low SNHG3 expression levels had a shorter overall survival compared with those with high SNHG3 expression levels (Figure 1(b)). Similar to the patient studies, SNHG3 expression levels were also found to be markedly downregulated in LUAD cell lines (A549, H1299, and H1975) compared with 16HBE cells (Figure 1(c)). The expression levels of SNHG3 were downregulated to the greatest extent in A549 and H1299 cells; therefore, these two cell lines were selected for use in subsequent experiments. These results indicated that SNHG3 expression levels may be significantly downregulated in LUAD tissues and cells.

### 3.2. SNHG3 Overexpression Inhibits the Proliferation, Migration, and Invasion, and Promotes the Apoptosis, of LUAD Cells

To determine the function of SNHG3 in LUAD, pcDNA3.1 SNHG3 vectors were transfected into A549 and H1299 cells. Following transfection, SNHG3 expression levels were markedly upregulated (Figure 2(a)). The results of the CCK-8 and colony formation assays demonstrated that SNHG3 overexpression inhibited the proliferation of LUAD cells (Figures 2(b) and 2(c)). In addition, flow cytometric analysis found that SNHG3 overexpression induced the apoptosis of LUAD cells (Figure 2(d)). To investigate the effects of SNHG3 on the migration and invasion of A549 and H1299 cells, wound healing and Transwell invasion assays were performed. The results of the wound healing assay revealed that the migration was decreased following the overexpression of SNHG3 in LUAD cells (Figure 2(e)). Similarly, the results of the Transwell assay demonstrated that SNHG3 overexpression inhibited the invasive abilities of LUAD cells (Figure 2(f)). These findings suggested that SNHG3 overexpression may inhibit the proliferation, migration, and invasion and promote the apoptosis of LUAD cells.

### 3.3. SNHG3 Directly Binds to miR-890 and Downregulates miR-890 Expression

To identify specific miRNAs modulated by SNHG3 in LUAD, downstream genes of SNHG3 were searched for using bioinformatics analysis. Data from The Cancer Genome Atlas database identified a potential binding site between SNHG3 and miR-890 (Figure 3(a)). Furthermore, a dual luciferase reporter assay was performed, and the results found that the cotransfection with the miR-890 inhibitor increased the relative luciferase activity of the SNHG3-Wt reporter vector compared with the cotransfection with the NC inhibitor. However, no significant differences were observed in the relative luciferase activity of the SNHG3-Mut reporter vectors between cells cotransfected with the miR-890 inhibitor or NC inhibitor (Figure 3(b)). In addition, SNHG3 overexpression was found to downregulate miR-890 expression (Figure 3(c)). Thus, the expression levels of miR-890 in LUAD tissues and cell lines were further analyzed. RT-qPCR analysis revealed that the expression levels of miR-890 were upregulated in LUAD tissues and cell lines (Figures 3(d) and 3(e)). These results indicated that miR-890 may be a target of SNHG3 and be negatively regulated by SNHG3.

### 3.4. SNHG3 Exerts Its Effects in LUAD by Regulating miR-890 Expression

To determine whether miR-890 was involved in promoting the effects of SNHG3 in LUAD, a miR-890 mimic was transfected into A549 and H1299 cells following the overexpression of SNHG3. The transfection efficiencies of the miR-890 mimic transfection and cotransfection of the miR-890 mimic and SNHG3 overexpression plasmid are presented in Figure 4(a). The expression levels of miR-890 were upregulated following the overexpression of miR-890, while the expression levels of miR-890 were downregulated following the overexpression of SNHG3. The results of the CCK-8 and colony formation assays demonstrated that miR-890 overexpression increased the proliferation of LUAD cells, while the SNHG3-overexpression-induced inhibition of LUAD cell proliferation was impaired following miR-890 overexpression (Figures 4(b) and 4(c)). Flow cytometric analysis showed that miR-890 overexpression inhibited the apoptosis of LUAD cells. Conversely, the increased apoptotic rate following SNHG3 overexpression was weakened following miR-890 overexpression (Figure 4(d)). The results of the wound healing and Transwell chamber assays showed that the migratory and invasive abilities of LUAD cells were increased following the overexpression of miR-890, while the inhibitory effects of SNHG3 overexpression on migration and invasion were partially antagonized by miR-890 overexpression (Figures 4(e) and 4(f)). Therefore, miR-890 overexpression promoted the progression of LUAD. SNHG3 activated LUAD progression by regulating miR-890.

## 4. Discussion

LUAD is one of the most common types of malignancy worldwide, accounting for high mortality rates [1, 2]. Therefore, determining the specific underlying mechanisms of LUAD remains a priority for the development of effective treatments for patients with LUAD. Currently, numerous studies have reported roles for and determined the underlying mechanisms of lncRNAs in LUAD [12–17]. In particular, the lncRNA SNHG3 was discovered to serve as a competing endogenous RNA to regulate the progression of various cancer types [18–20]. For example, SNHG3 promoted hepatocellular tumorigenesis by regulating miR-326 expression [21], and SNHG3 modulated the miR-384/WEE1 G_2_ checkpoint kinase axis to regulate laryngeal carcinoma cell proliferation and migration [22]. In addition, the lncRNA SNHG3 was reported to play a vital role in LUAD progression [23, 24]. However, to the best of our knowledge, the tumorigenic properties and underlying mechanism of action of SNHG3 in LUAD progression remain to the determined. The present study characterized the expression pattern and molecular mechanism of SNHG3 in LUAD. The expression levels of SNHG3 were found to be downregulated in both clinical samples from patients with LUAD and LUAD cell lines. Furthermore, SNHG3 overexpression inhibited the proliferation, migration, and invasion and promoted the apoptosis of LUAD cells, which indicated that SNHG3 may regulate the malignant behavior of LUAD cells by serving as an oncogene in LUAD. Mechanistically, SNHG3 promoted LUAD progression by regulating miR-890 expression.

An increasing number of studies have demonstrated that miRNAs exert both tumor suppressive and oncogenic roles in tumorigenesis, and the expression of lncRNAs can regulate the activities of miRNAs [25, 26]. Therefore, miRNAs have shown promise as potential clinical biomarkers and therapeutic targets for the treatment of patients with LUAD [27–29]. To date, numerous studies have revealed that miR-890 was associated with the progression of a large number of cancer types [30, 31]. For instance, miR-890 repressed the proliferation and invasion and induced apoptosis in breast cancer cells by regulating CD147 expression [32]. Nevertheless, to the best of our knowledge, the functional role of miR-890 in the evaluation of LUAD status remains unclear. Based on the results of a previous study, the present study further investigated the function of miR-890 in LUAD development. Using bioinformatics analysis and a dual luciferase reporter assay, SNHG3 was predicted to directly bind to miR-890. Moreover, miR-890 expression was negatively regulated by SNHG3, and miR-890 expression levels were found to be upregulated in both LUAD tissues and cell lines. In addition, miR-890 overexpression promoted the proliferation, migration, and invasion and inhibited the apoptosis of LUAD cells. Thus, miR-890 overexpression abrogated the effects of SNHG3 overexpression on LUAD cells. Thus, it is suggested that SNHG3 may promote the occurrence and progression of LUAD by regulating miR-890 expression.

Nonetheless, there are several limitations to the present study. First, although there are a large number of lncRNAs, the current study only determined the role of lncRNA SNHG3 and miR-890 in LUAD. Second, the study did not investigate the association between other lncRNAs and lung cancer and any other potential interactions between genes. Therefore, future studies will focus on the interactions between lncRNAs.

In conclusion, to the best of our knowledge, the current study was the first to report the function and regulatory mechanism of the lncRNA SNHG3 in LUAD. The findings suggested that SNHG3 may function as an oncogene in LUAD by modulating the expression levels of miR-890. Therefore, lncRNA SNHG3 and miR-890 may serve as novel biomarkers or potential targets for the treatment of LUAD.

## Figures and Tables

**Figure 1:** The SNHG3 expression is downregulated in LUAD tissues and cell lines. (a) Relative expression levels of lncRNA SNHG3 in LUAD tissues and normal tissues were detected by RT-qPCR. ^*∗*^*P* < 0.05 vs. the normal tissue. (b) The GEPIA database was used to evaluate the relationship between SNHG3 expression and the prognosis of LUAD patients with overall survival (OS). (c) Relative expression levels of lncRNA SNHG3 in different LUAD cell lines were detected by RT-qPCR. ^*∗*^*P* < 0.05, ^*∗∗*^*P* < 0.01 vs. the normal tissue the 16HBE cell line.

**Figure 2:** SNHG3 overexpression inhibits the progression of LUAD cells. (a) The transfection efficiency of pcDNA3.1 SNHG3 was verified by RT-qPCR assay. (b) Cell viability was detected by CCK-8 assay. (c) Cell proliferation was detected by clone formation assay. (d) Cell apoptosis was determined by flow cytometry assay. (e) Cell migration was detected by wound scratch assay. (f) Cell invasion was detected by transwell chamber assay. ^#^*P* < 0.05, ^*∗∗*^*P* < 0.01 vs. blank and pcDNA3.1.

**Figure 3:** SNHG3 directly binds to miR-890 and downregulates the miR-890 expression. (a) The putative miR-890 binding sites for SNHG3. (b) Luciferase reporter assay was applied to assess the relationship between SNHG3 and miR-890. ^*∗*^*P* < 0.05 vs. blank and NC-inhibitor. (c) Relative mRNA expression level of miR-890 was detected by RT-qPCR when cells were transfected with pcDNA3.1 SNHG3. ^*∗*^*P* < 0.05 vs. blank and pcDNA3.1. (d) Relative expression levels of miR-890 in LUAD tissues and normal tissues were detected by RT-qPCR. ^*∗∗*^*P* < 0.01 vs. the normal tissue. (e) Relative expression levels of lncRNA SNHG3 in different LUAD cell lines were detected by RT-qPCR. ^*∗*^*P* < 0.05, ^*∗∗*^*P* < 0.01 vs. the normal tissue the 16HBE cell line.

**Figure 4:** SNHG3 promotes the progression of LUAD by regulating miR-890. (a) The relative expression level of miR-890 in A549 and H1299 cells transfected with miR-890 mimic and pcDNA3.1 SNHG3+miR-216a-3p mimic was measured by RT-qPCR. (b) Cell viability was detected by CCK-8 assay. (c) Cell proliferation was detected by clone formation assay. (d) Cell apoptosis was determined by flow cytometry assay. (e) Cell migration was determined by wound healing assay. (f) Cell invasion was determined by transwell chamber assay. ^*∗*^*P* < 0.05, ^*∗∗*^*P* < 0.01 vs. blank and NC mimic.

**Table 1:** The expression of SNHG3 and clinicopathological features in 66 lung adenocarcinoma. ^*∗*^*P* values are calculated with the chi-square test.

Clinicopathological features	Cases (*n* = 66)	SNHG3 expression		*P* value^*∗*^
		38 high (%)	28 low (%)	

Gender				
Male	34	20 (58.8)	14 (41.2)	0.833
Female	32	18 (56.3)	14 (43.8)	

Age (years)				
≤60	33	17 (51.5)	16 (48.5)	0.319
>60	33	21 (63.6)	12 (36.4)	

Tumor size (mm)				
≤5.0	39	24 (61.5)	15 (38.5)	0.434
>5.0	27	14 (51.9)	13 (48.1)	

TNM stage				
I-II	38	27 (71.1)	11 (28.9)	0.010^*∗*^
III-IV	28	11 (39.3)	17 (60.7)	

Lymph node metastasis				
0–2	41	29 (70.7)	12 (29.3)	0.014^*∗*^
>2	25	11 (40.7)	16 (59.3)	

## Data Availability

The simulation experiment data used to support the findings of this study are available from the corresponding author upon request.
